# Relationship between Intestinal Microflora and Hepatocellular Cancer Based on Gut-Liver Axis Theory

**DOI:** 10.1155/2022/6533628

**Published:** 2022-08-01

**Authors:** Shipeng Li, Wenfeng Han, Qichen He, Wei Zhang, Youcheng Zhang

**Affiliations:** ^1^Department of General Surgery, Lanzhou University Second Hospital, Lanzhou, China; ^2^Department of Surgical Oncology, Gansu Provincial Cancer Hospital, Lanzhou, China; ^3^Lanzhou Hospital of Traditional Chinese Medicine, Lanzhou, China

## Abstract

The intestinal microflora is a bacterial group that lives in the human digestive tract and has a long-term interdependence with the host. Due to the close anatomical and functional relationship between the liver and the intestine, the intestinal flora affects liver metabolism via the intestinal-hepatic circulation, thereby playing an extremely important role in the pathological process of liver inflammation, chronic fibrosis, and liver cancer. In recent years, the rapid development of technologies in high-throughput sequencing and genomics has opened up possibilities for a broader and deeper understanding of the crosstalk between the intestinal flora and the occurrence and development of liver cancer. This review aims to summarize the mechanisms by which the gut microbiota changes the body's metabolism, through the gut-liver axis, thereby affecting the occurrence and development of primary liver cancer. In addition, the potential regulation of intestinal microflora in the treatment of liver cancer is discussed.

## 1. Introduction

Hepatocellular cancer (HCC) is one of the most common malignant tumors of the digestive system. According to global cancer statistics, there were 905,677 new cases of HCC and 830,180 deaths worldwide in 2020, and over 50% of new cases and mortality of HCC patients occurred in China [1, 2]. HCC is mainly believed to be related to drinking alcohol or long-term chronic liver disease (CLD), such as fatty liver, cirrhosis, chronic hepatitis (hepatitis B virus (HBV) and hepatitis C virus (HCV) infection), autoimmunity, cholestasis, smoking, diabetes, and obesity [3–5]. In recent years, it has been shown that the intestinal flora is closely related to HCC. Firstly, the intestinal flora can promote the development of HCC through various mechanisms. Secondly, the efficacy and adverse effect of HCC tumor immunotherapy are also related to the intestinal flora, especially impacting the effects of immunosuppressive agents [6]. Due to the bidirectional communication between the intestine and the liver, on the one hand, the liver excretes bile acid and other biologically active components through the bile duct to communicate with the intestine; on the other hand, the metabolic nutrients absorbed by the intestine are transported to the liver through the portal vein. Intestinal bacteria and their products, endotoxins and inflammatory mediators, will also be transported to the liver through the portal vein, making the liver susceptible to pathological changes of the intestinal microenvironment [7]. The gut-liver axis theory facilitates a better understanding of the crosstalk between intestinal flora and liver diseases.

## 2. The Composition of the Intestinal Microflora

In normal physiological conditions, about 500–1000 different bacteria are colonized in the human intestine, with a total weight of more than 1 kg, most of which are anaerobic. There is a specific symbiotic relationship between them and the human body. They participate in digestion, vitamin synthesis, and immune regulation; promote angiogenesis; regulate nerve function; and maintain the body's homeostasis, playing a key role in the body's physiology and pathology [8]. In physiological conditions, the intestinal microflora resides in the intestine in a relatively stable manner, but it is easily affected by the internal and external environmental factors, such as diet, drinking, smoking, drugs, obesity, genetics, and digestive tract diseases. Disturbance of the homeostasis of intestinal flora leads to a series of pathological changes.

The intestinal flora is basically composed of five phyla, namely, Firmicutes, Bacteroidota, Actinobacteria, Proteobacteria, and Verrucomicrobia, among which Firmicutes (79.4%) and Bacteroidota (16.9%) dominate the intestinal flora of healthy adults and play an important role in providing energy and nutrition to the host [9]. Firmicutes, Bacteroidota, and Bifidobacteria play a synergistic role, that is, using indigestible carbohydrates to generate SCFAs [10]. There are also a small amount of *Lactobacillus*, *Streptococcus*, and *Escherichia coli* in the intestine. Colonization of these bacteria can induce goblet cell differentiation and mucus production, which can inhibit *Salmonella typhimurium*, pathogenic *Escherichia coli*, *Clostridium difficile*, etc., contributing to epithelial cell function and energy balance.

## 3. Gut-Liver Axis

Due to the unique anatomical and functional relationship between the gastrointestinal tract and the liver, the gut-liver axis through the portal vein becomes the most important two-way communication between the gut microbiota and the liver. Approximately 70% of the blood supply of the liver comes from the intestinal tract. Usually, the nutrients digested and absorbed by the intestine, such as glucose, lipids, proteins, and vitamins, and bacteria and bacterial components such as lipopolysaccharide (LPS) and other intestine-derived factors circulate through the portal vein to the liver. When the intestinal barrier is damaged, its permeability increases and the liver will be insulted by a variety of toxic agents from intestine and harmful intestinal bacteria. The imbalance of intestinal flora may aggravate this process [11]. The core of a healthy gut-liver axis lies in a fully functioning intestinal mucosal barrier, which is directly related to the balanced intestinal flora. The mechanical connection between intestinal epithelial cells is a natural barrier for bacteria and their metabolites. However, it is not a static physical barrier, but the result of an interaction between the intestinal flora and immune cells, which includes antigen-specific immune response, immune balance, and tolerance.

The intestinal barriers include mechanical barriers, chemical barriers, immune barriers, and biological barriers. They are mainly composed of intact intestinal mucosal epithelia, intestinal mucus, Paneth cells, goblet cells, mucosa-associated lymphoid tissues, and many secreted factors such as immunoglobulin A(IgA) or defensins [12]. The intestinal barrier can effectively prevent harmful intestinal bacteria and their metabolites from entering the circulation to cause bacteremia or other tissue damage. Changes in the intestinal barrier are the driving factors of inflammation and will significantly affect the gut-liver axis. By preventing direct contact between the bacteria and epithelial cells, the mucosal layer of the intestinal barrier is the first-line defense when external molecules reach the intestinal lumen [13]. The intestinal barrier and the intestinal flora can also influence each other. On the one hand, intestinal cells can regulate the intestinal flora by secreting antimicrobial peptides. On the other hand, the growth of the intestinal barrier and intestinal epithelial cells can also be affected by the intestinal flora. In addition, the intestinal flora can also inhibit the growth of pathogenic microorganisms, thereby maintaining the homeostasis of intestinal microorganisms. Although the intestinal barrier shields the liver from exposing to a large amount of proinflammatory microbial-associated molecular patterns, acute and chronic liver diseases often affect the composition of the intestinal flora and the function of the intestinal barrier, leading to imbalance of the intestinal flora and intestinal leakage. These effects may be harmful, for instance, activating the liver immune response and releasing proinflammatory cytokines to aggravate liver damage; sometimes, they may be beneficial, such as strengthening cell protection and promoting liver cell regeneration. It is worth mentioning that not only is the liver affected by the input of intestinal microbes, but in turn, it can also affect the intestinal microbes via secreting bile acids, IgA antibodies, and other metabolites. Therefore, the liver plays an important role in the regulation of microbial remodeling [8].

## 4. Intestinal Flora and HCC

HCC occurs almost exclusively in patients with chronic liver disease and is driven by a vicious cycle of liver damage, inflammation, and regeneration that often spans decades.

Therefore, liver fibrosis and cirrhosis may lead to HCC [2]. In the human body, intestinal microbes interact with the host through the gut-liver circulation and microecological-liver axis, which are involved in the initiation and development of liver inflammation, chronic fibrosis, and cirrhosis [7]. According to statistics, about 80%∼90% of HCC cases have advanced liver fibrosis or cirrhosis. In addition, about 5%∼25% of patients with cirrhosis will eventually develop into HCC.

### 4.1. Intestinal Flora and Chronic Liver Disease

Chronic liver disease may progress to HCC. The chronic inflammation underlying alcoholic hepatitis, nonalcoholic steatohepatitis, and chronic hepatitis might be the driving factor of HCC. Bacterial components from the intestine are stimulators for liver inflammation through the gut-liver axis. The proinflammatory role of intestinal bacterial compounds is regulated by Toll-like receptors. The inflammatory mediators produced by various pathways can promote the aggregation, proliferation, and activation of Kupffer cells, neutrophils, and hepatic stellate cells. Activation of these cells produces more inflammatory mediators, like chemokines and reactive oxygen species that could cause liver cell damage. Suppression of the intestine flora by antibiotics could diminish liver inflammation and damage [14]. The study of Lin et al. [15] confirmed that in the process of acute hepatitis induced by concanavalin A in rats, elimination of intestinal microecology enhanced the effect of LPS and Toll-like receptor 4 (TLR4) on Kupffer cells. Activation of TLR4 stimulates subsequent inflammatory signaling pathways and aggravates hepatitis induced lesions.

### 4.2. Intestinal Flora and Liver Fibrosis

There is a strong correlation between liver fibrosis and development of HCC. Liver fibrosis is an important risk factor for the development of HCC. Rodriguez et al. [16] showed that compared with the healthy control group, the intestinal flora of the liver fibrosis group was imbalanced, manifested as changes in the content of Verrucomicrobia, *laevis*, actinomycetes, *Desulfovibrio*, and *Lactobacillus*. The abundance of bacilli and bifidobacteria was significantly increased. As a probiotic, abundance of Verrucomicrobia is positively correlated with gastrointestinal health. Inhibition of the intestinal flora by antibiotics prevents liver damage and fibrosis caused by carbon tetrachloride or choline deficiency diet, while the endotoxin from intestinal flora increases liver fibrosis caused by choline deficiency diet [17]. Another study [18] showed that in sterile mice, intestinal sterilization increases liver fibrosis, indicating contradictory effect of antibiotics on liver fibrosis. Endogenous symbiotic microbiota offers hepatic protection signals, since the complete removal of the intestinal flora (sterile mice) can increase liver damage. These phenomena may be due to the activation of antiapoptotic NF-*κ*B signaling pathway mediated by the absence of TLR4, subsequently aggravating liver fibrosis.

### 4.3. Intestinal Flora and Liver Cirrhosis

In liver cirrhosis, due to decreased immune function, slow bowel movement, hypoproteinemia, portal hypertension, and other factors, the mesenteric ischemia and intestinal motility are downgraded, leading to decreased beneficial bacteria such as *Bacteroidota* and *Clostridium* and increased invasion and colonization of conditional pathogenic bacteria such as *Enterobacter* and *Veillonella* spp., finally resulting in imbalanced intestinal flora. Chen et al. [19] found that the structure of the intestinal flora of patients with liver cirrhosis was significantly different from that of healthy controls, and the degree of intestinal microecological imbalance was positively correlated with the severity of liver cirrhosis. In the fecal flora, the phylum of Bacteroidota in patients with cirrhosis was significantly reduced compared with healthy individuals, while the phyla of Proteobacteria and Fusobacteria were significantly increased, accompanied by an increase in potentially pathogenic Enterobacteriaceae, *Veronococcus*, and *Streptococcus*. Qin et al. [20] also verified this change through metagenomics research and analysis, and it was found that 54% of the intestinal flora of patients with liver cirrhosis originated from the oral cavity, thereby proposing the hypothesis that the oral flora invaded the gastrointestinal tract in patients with liver cirrhosis. In addition, other studies [21–23] indicate that imbalanced intestinal flora plays a key role in the pathophysiological process of the occurrence and development of liver cirrhosis-related complications, such as spontaneous bacterial peritonitis and hepatic encephalopathy.

## 5. The Mechanism of Intestinal Flora Involvement in the Occurrence and Development of Liver Cancer

In recent years, more and more evidence has confirmed that the imbalance of intestinal flora plays an important role in the occurrence and development of liver cancer [24–27]. In addition to the differences in the types of microbial components and the intuitive changes in the amount of the intestinal flora in HCC patients, it is also necessary to explore the impact of its metabolites on the liver, flora migration, destruction of the intestinal barrier, and participation in immune response.

### 5.1. The Imbalance of the Intestinal Flora Promotes the Development of HCC

The imbalance of the flora often plays a key role in the development of chronic liver disease and HCC. The imbalance of the flora is mainly driven by the pathological conditions of end-stage liver disease, such as decreased bile secretion, changes in antimicrobial peptides, and IgA secretion by the intestinal tract. It has been found that the main manifestations of the imbalance of the flora in patients with chronic liver disease and cirrhosis are increased potential pathogenic bacteria, decreased beneficial bacteria, and translocation of the flora from the gut to the liver. Imbalanced intestinal flora weakens the colonization resistance of itself and loses the barrier protection role, triggering colonization and invasion of other potential pathogens (including conditional pathogens) in the intestine. For instance, a high-fat diet causes an increase in Gram-negative bacteria in the intestine of mice, while decreasing the ratio of *Bacteroidota* to scleroderma. In addition, it has been shown that flora imbalance is transmissible in the occurrence and development of liver diseases. For example, transplanting imbalanced intestinal flora to mice on a controlled diet increases liver damage and fibrosis. Although there is no direct evidence indicating that the transmission of flora can increase the risk of HCC, mice inoculated with probiotics before tumor cell inoculation can inhibit the formation of HCC [28, 29].

Intestinal bacterial components can not only directly cause liver inflammation, but also regulate the immune system to trigger inflammation. The immune system recognizes MAMPs through the pattern recognition receptors (PRRs), such as TLR4 and nucleotide oligomerization region-like receptors (NLRs) [14, 30]. Toll-like receptor (TLR) is a protein that plays an important role in the crosstalk between nonspecific immunity (natural immunity) and specific immunity (acquired immunity). When the body's physical barriers (skin, mucous membranes, etc.) are challenged by microorganisms, TLR will recognize these microorganisms and stimulate the immune response. KCs, HSCs, and hepatocytes in the liver express TLR4, which can recognize LPS from the intestinal flora. Activation of TLR4 by LPS regulates the expression levels of other immune molecules through a series of responses. Activation of TLR4 in HSCs will lead to upregulation of NF-*κ*B-mediated hepatic mitogen activated protein and promote mitosis of hepatocytes. On the other hand, activation of LPS-TLR4 axis leads to NF-*κ*B-mediated hindrance of hepatocyte apoptosis, which ultimately promotes the formation of liver cancer. KCs in the liver secrete inflammatory cytokines such as TNF-*α* and IL-6 in large quantities during LPS-TLR4 activation, causing oxidative stress and inflammation in the liver, eventually damaging cell DNA and leading to gene mutations [14, 31]. Meanwhile, HSCs in the liver are activated by the LPS-TLR4 pathway to synthesize and secrete excessive extracellular matrix proteins, promoting the occurrence and development of liver cirrhosis. LPS activated HSCs also secrete angiogenic factors, promoting migration of mesenchymal endothelial cells and blood vessels formation, which is a key step in promoting the progression of HCC.

In addition, it has been shown that the TLR4 signaling pathway of tumor cells is basically the same as that of immune cells. In particular, tumor cells use TLR4 expressed on their surface to maintain a microenvironment that is conducive to tumor cell survival, thereby evading the body's immune attack [32]. Clinical studies have confirmed that the expression of TLR4 in HCC patients is closely related to liver cancer metastasis, early recurrence, and poor survival. The activation of TLR4 by LPS in liver cancer cell lines enhances their invasion ability and epithelial-mesenchymal transition and promotes the occurrence of HCC, suggesting that TLR4 may be a practical biological indicator of liver cancer metastasis and recurrence. Yu and Schwabe [14] first comprehensively explained the role of intestinal-derived LPS in the occurrence of HCC. Their study found that intestinal sterilization and downregulation of TLR4 can reduce the incidence of liver tumors and inhibit tumor growth. In addition, it was revealed that TLR4 is a tumor stem cell marker, whose abnormal expression induces stem cell-like characteristics by activating the TLR4/Nanog pathway [33, 34]. Therefore, targeting TLR4 or its homologous signals might be a potential molecular target for HCC treatment by regulating the proliferation and chemotherapy sensitivity of liver cancer cells.

In addition to TLR4, the activation of TLR2 also promotes the occurrence of hepatocytes. A study [35] showed that lipoteichoic acid (LPA) and deoxycholic acid in the intestinal flora can upregulate senescence-related secreted phenotype (SASP) factors through Toll-like receptor 2 (TLR2) expressed on hepatic stellate cells and enhance the expression of COX2 molecules. Furthermore, COX2-mediated prostaglandin 2 (PGE2) inhibits antitumor immunity through the prostaglandin EP4 receptor (PTGER4), thereby promoting the development of HCC. In addition, intestinal flora and its components affect cell differentiation. For instance, LPS increases hepatocyte proliferation through TLR4, thereby increasing the risk of HCC. Inoculating mice with probiotics can inhibit the differentiation of Th17 cells and reduce the secretion of IL17, decreasing the occurrence and development of liver cancer [36].

### 5.2. The Imbalance of the Metabolites of Intestinal Flora Promotes the Development of HCC

Intestinal bacterial components, such as LPS, polypeptides, and bacterial DNA, enter the mesenteric lymph nodes or other extraintestinal organs through the intestinal mucosal barrier. When the liver is damaged, Kupffer cells (KCs) are affected by these components. The internal pericytes are inhibited, and the elimination of endotoxin is weakened. In addition, the continuous portal hypertension opens the portal-caval collateral circulation, resulting in high levels of endotoxemia in the hepatic circulation and causing chronic liver inflammation [37]. When the intestinal flora is imbalanced and the intestinal bacteria overgrow, bacterial components (especially LPS) are increased greatly and the intestinal barrier function is significantly reduced. As a result, a large amount of LPS enters the liver through the portal vein and activates TLR4 expressed on KCs, hepatic stellate cells (HSCs), and liver cancer cells, promoting chronic hepatitis, cirrhosis, and even liver cancer [38]. Intestinal metabolites can not only aggravate the liver damage that has been formed, but also induce systemic metabolic and hemodynamic disorders, thus forming a vicious circle that continues to aggravate liver diseases. There is evidence that the malignant degree of abnormal liver function is related to the level of LPS and other bacterial substances. High concentrations of LPS and other bacterial substances in the blood can cause liver cell damage, deteriorating liver fibrosis [37]. In addition, LPS induces the secretion of a variety of inflammatory factors, such as TNF-*α*, IL-6, and TGF-*β*, which are involved in liver disease caused by LPS, especially in the end-stage liver disease, such as hepatitis B or C virus infection induced liver cancer [39].

Bile acid is an important component of bile and a metabolite of cholesterol, which is mainly present in the enterohepatic circulatory system. Intestinal microbes interact with bile acid. Bile acid shapes the intestinal microbial community. In turn, intestinal microbes can change the storage of bile acid. Studies have shown [40–42] that high concentration of bile acid which exceeds the physiological range may cause cytotoxicity, inducing cell necrosis. Bile acid and liver disease are closely related. Bile acids act on bile acid-related receptors to regulate liver physiology. Bile acid-related pathological research in liver is even trendier. At present, most studies on bile acid receptors focus on farnesoid receptors (FXR), transmembrane G protein-coupled receptor 5 (TGR5), and CXCR6, to explain the mechanism of bile acid and its receptors in the liver disease development. Homeostasis of bile acid and interaction with its receptor are closely related to immune response, cell proliferation, and apoptosis.

FXR, mainly distributed in liver and small intestine tissues, is the main regulator of bile acid balance and enterohepatic circulation, and bile acid is its natural ligand. When the intestine is in an environment with a high level of bile acid, intestinal FXR is activated. Both free bile acid and bound bile acid can activate FXR. The latter inhibits the rate-limiting enzyme of bile acid synthesis, CYP7A1, whose transcription mediates the negative feedback regulation of bile acid synthesis. The activated FXR stimulates intestinal hormone fibroblast growth factor 15/19 (FGF15/19), which binds to corresponding receptors on the surface of hepatocytes, inhibiting the transcription of CYP7A1 gene. FGF15 can be used as a secondary or auxiliary mitogen for hepatocytes and enhances the growth of hepatocyte primary mitogens, leading to mitogenic effects, such as increasing hepatocyte growth factor and epidermal growth factor. Therefore, the intestinal bile acid/FXR/FGF15 signaling axis promotes liver regeneration with bile acid overload [43–45]. Activated FXR also inhibits the uptake and promotes the secretion of bile acid by regulating the expression of bile acid transporters in the liver and intestine, thereby inhibiting the accumulation of bile acid in hepatocytes and ensuring the stability of bile acid storage in the enterohepatic circulation and intestinal cavity.

TGR5 is a bile acid membrane receptor, expressed in biliary and intestinal epithelial cells and immune cells. TGR5 can be activated by a variety of bile acids, thereby affecting the homeostasis of bile acids. Stimulation of TGR5 in the liver and intestine inhibits the expression and secretion of cytokines, which can reduce the transcriptional activity of NF-*к*B, thereby reducing liver and intestinal inflammation, preventing chronic hepatitis, and abating the occurrence and development of liver disease [46, 47]. While activation of TGR5 has many protective effects, it may also lead to deleterious outcomes. Due to its pro-proliferative and antiapoptotic properties, it is closely related to the pathogenesis of hepatocellular carcinoma and cholangiocarcinoma [48].

In recent years, CXCR6 has gradually become a target for the treatment of HCC by mediating innate immunity in the liver [49–51]. The intestinal microbiota utilizes bile acid as messengers to regulate the level of chemokine CXCL16 in hepatic sinusoidal endothelial cells, thereby regulating the accumulation of CXCR6 hepatic natural killer cells (NKT cells). The accumulated NKT cell is a highly activated phenotype, and the antigen stimulates INF- *γ* level, thereby inhibiting the growth of liver cancer. The result of an animal experiment suggested that modulation of intestinal commensal bacteria can specifically alter the growth kinetics of liver tumors. Compared to controls, in mouse models with inhibited intestinal bacterial growth, there were not only more hepatic NKT cells, but also activated NKT cells. The number of surviving and aggregated CXCR6+ cells was also increased, which inhibited the growth, spread, and metastasis of liver cancer cells [52].

## 6. The Role of Intestinal Flora in the Prevention and Treatment of Liver Cancer

Currently, there are many available treatments for HCC. In addition to surgery, chemotherapy and radiotherapy, transcatheter hepatic artery embolization, hepatic artery infusion chemoembolization, molecular targeting, and immunotherapy are also available. Although the treatments are effective to a certain extent, there have also been significant complications and adverse effects. In recent years, with an increased number of studies on liver diseases caused by intestinal flora imbalance, targeted intestinal flora regulation may become a new way to treat or prevent the development of HCC.

### 6.1. Application of Probiotics in the Prevention and Treatment of HCC

Probiotics are a class of active microorganisms that are beneficial to the human body, including *Lactobacillus* and *Bifidobacterium*, which can improve the intestinal microecology. More and more studies have found that probiotics play a unique role in preventing the onset of HCC: (1) Probiotics can improve the intestinal microecology, protect the mucosal barrier, and reduce the activation of the LPS-TLR4 pathway by modeling bacterial components (especially LPS), thereby preventing the occurrence of HCC. It was found [53] that high-dose *Lactobacillus* LF41 improved intestinal and liver innate immunity in normal mice. After 10 days of treatment in the digestive tract of normal mice, it was found that the expression levels of COX-2 and IL-10 in ileum and PGE2 in the liver were significantly increased, which promoted the expression of IL-10 in the liver mediated by LPS, facilitating resistance to LPS-induced liver injury and expression of TNF-*α*. Since both liver inflammation and cirrhosis can cause HCC, probiotics play an active role in the treatment of liver inflammation and cirrhosis and could effectively prevent liver cancer. (2) Probiotics can also reduce carcinogenetic effects and prevent HCC. Recently, it is reported that *Bacillus subtilis* can degrade aflatoxin, while the probiotic compound made from *Bacillus subtilis*, *Lactobacillus casei*, and *Candida utilis* has a higher degradation rate. This suggests that probiotic formulations can reduce the exposure dose of aflatoxin and have a positive effect on the prevention of HCC [54]. In addition, it has been shown that probiotic mixtures increase the expression of tight junction proteins by activating p38 and ERK signaling pathways, protecting the intestinal epithelial barrier, and preventing bacterial products such as endotoxins from entering the portal circulation from the intestine [55]. (3) Probiotics also improve the innate immunity of the liver and intestine, thereby enhancing clearance of hepatitis viruses by the liver, reducing liver inflammation and strengthening the intestinal barrier function, ultimately exerting an anticancer effect [56–58]. It has been shown that, on the one hand, probiotics may stimulate the secretion of anti-inflammatory substances by *Prevotella*; on the other hand, probiotics may effectively suppress the development of HCC by inhibiting IL-17 secretion in tumors. This subset of helper T cells can inhibit tumor immunity, stimulate tumor angiogenesis, and participate in the occurrence and development of tumors [56].

### 6.2. Fecal Microbiota Transplantation

Fecal microbiota transplantation (FMT) refers to a process of introducing the fecal flora suspensions from healthy donors into the gastrointestinal tract of patients to reconstruct the microecological structure and function of the intestinal flora [59]. A preliminary clinical trial using FMT from healthy donors for the treatment of severe alcoholic hepatitis found that markers associated with liver disease severity (total bilirubin, Child–Pugh score, and end-stage liver disease score) were significantly improved within 1 week of FMT treatment [60]. Iida [61] found that the intestinal flora can modulate the therapeutic effect of tumors by regulating the tumor microenvironment. HCC is a chronic liver disease, and the use of FMT is a very attractive prevention strategy. FMT is effective in the treatment of chronic liver disease and may play a role by restoring intestinal microecological balance in patients. Some studies have also shown that FMT is also beneficial to the delay of the progression of HCC; however, solid evidence is lacking due to too few relevant studies. In addition, we should also fully consider the safety of FMT therapy. Future studies on clarification of active ingredients with the therapeutic effect of FMT are needed to reduce the infection of unknown pathogens caused by FMT, increasing the safety of treatment for the HCC patients through regulating the intestinal microecology.

### 6.3. Antibiotics

Antibiotics can prevent the translocation of intestinal microbes and their metabolites, reduce intestinal microbial load, and improve the balance of intestinal flora. It was reported that penicillin or sodium dextran sulfate induced intestinal flora imbalance and significantly promoted the development of HCC in mice; probiotics restored the balance of intestinal flora, not only reducing the plasma lipopolysaccharide level, but also reducing the number and volume of tumors in mice [29]. Huynh et al. [62] used bevacizumab combined with rapamycin to inhibit the growth of HCC, which was significantly better than monotherapy and markedly prolonged the survival time of HCC mice. It is noteworthy that, on the one hand, antibiotics can inhibit the inflammatory response caused by harmful intestinal flora and reduce the incidence of chronic hepatitis or HCC. On the other hand, long-term abuse of antibiotics can also lead to the disturbance of the originally complex intestinal microecological balance, triggering other diseases or accelerating the progression of the disease.

### 6.4. Traditional Chinese Medicine

Traditional Chinese medicine (TCM) and its ingredient compounds are complex, being able to act on the “gut-liver axis” via multiple targets and links and at multiple levels. Intestinal microbes and active ingredients of TCM have bidirectional regulatory effect. Specifically, the structure of the intestinal microbial composition is disordered. A series of inflammatory reactions can be normalized with the action of the active ingredients of TCM, and intestinal microorganisms are involved in the metabolism of the ingredients of TCM [63]. TCM can prevent and treat HCC by intervening related signal pathways, including Hedgehog signal pathway, IL-6/STAT3 signal pathway, NF-*к*B signal pathway, PI3K/Akt/mTOR signal pathway, MAPK signal pathway, TLR signal pathway, and Wnt signaling pathway [64–66]. At present, TCM is effective in preventing and treating HCC to a certain degree, but the specific mechanism has not been fully elucidated, and the signaling pathways involved remain to be explored.

## 7. Conclusions

As previously mentioned, the imbalance of the intestinal microecology may contribute to the development of HCC. However, there is no direct evidence of its role in human HCC. Therefore, it is necessary to further investigate the possible link between the intestinal flora and human HCC. Current studies have clarified that HCC patients, especially those with liver cirrhosis, have imbalanced intestinal flora, which will further aggravate the development of HCC and form a vicious circle. Appropriate modulation of the intestinal flora can be beneficial to the prevention and treatment of HCC. The mechanism behind the relationship between gut microbial components and HCC has been the focus of researchers in recent years. The development and application of new drugs based on corresponding targets have been discovered. However, they lack specificity for HCC. In addition, their targets on liver cancer cells are still not clear. It is unclear whether ligand-modified carriers can be developed as auxiliary targets for HCC cells. Moreover, there are differences in intestinal bacteria between different liver diseases, stages, and individuals. Whether these differences can be used as the criteria for liver disease classification and staging is unclear, which remains to be clarified by more studies.

## Data Availability

The datasets used and analyzed during the current study are available from the corresponding author upon reasonable request.
